# Study on the Mental Health of the Elderly under Different Pension Models

**DOI:** 10.1155/2022/2367406

**Published:** 2022-02-08

**Authors:** Jun Song, Lei Yang, Mingfei Han, Ying Wu

**Affiliations:** Shanghai Urban Construction Vocational College, Shanghai 201415, China

## Abstract

**Objective:**

To compare the mental health status of the elderly under different pension modes and to provide evidence for improving institutional services and the quality of life of the elderly.

**Methods:**

A total of 118 elderly people in social welfare homes, nursing homes, and elderly welfare centers in D city and 165 elderly people from families in D city were assessed by self-made questionnaire, Geriatric Depression Scale (GDS), activities of daily living scale (ADL), and social support rating scale (SSRS).

**Results:**

The total scores of mental health and self, emotion, and adaptation subscales in the social group were higher than those in the home group, with a significant difference (*p* > 0.05). The scores of cognitive and interpersonal subscales in the home group were higher than those in the social group, but the differences were not significant (*p* > 0.05). Under the mode of family pension and social institution pension, the health status of the elderly has certain differences. The elderly in different old-age care modes have good performance in diet and sleep, and there is no statistical difference between them (*p* > 0.05).

**Conclusion:**

The investigation shows that the mental health status of the elderly under the family pension model is obviously better than that under the social institution pension model.

## 1. Introduction

China has entered a period of rapid development of population aging and aging. In 2009, the number of elderly people over 60 years old in China reached 167 million, accounting for 12.5% of the total population [1]. It is predicted that the elderly population will reach 374 million by 2040, accounting for 24.48% of the total population [2]. At present, there are some social institutions for the aged, and there are more and more district-run, township-run, or private-run institutions for the aged, which pay more attention to the living care and physical health of the elderly, but pay little attention to their mental health and psychological needs. There have been some research studies on the mental health status and psychological needs of the elderly, but there are few research studies on the elderly under different pension modes [3].

This study summarizes the research progress of mental health status of the elderly under different pension modes. It is pointed out that the four pension modes of family pension, institutional pension, home pension, and mutual pension have their own advantages and disadvantages. Each mode should learn from each other and develop in a diversified way to jointly improve the mental health level and quality of life of the elderly. The state, society, and families should choose different pension modes according to the different ages, periods, and health states of the elderly and change the mode of one person into the mixed pension track of one person and multiple modes, so as to promote the vigorous development of pension undertakings in China.

Through the questionnaire, this study investigates the mental health status of the elderly under different pension modes, analyzes some existing problems, and puts forward some suggestions, hoping to arouse the attention of society, families, and the elderly themselves to the mental health of the elderly and at the same time provide scientific basis for the development and improvement of the pension cause.

## 2. Object and Methods

### 2.1. Object of Study

1. The social institution endowment group (social group) is the old people who provide for the aged in nursing homes, apartments for the elderly, and social welfare homes. A random questionnaire survey was conducted in more than 10 old-age care institutions at all levels, such as social welfare homes, nursing homes, and welfare centers for the elderly in D city, and 130 questionnaires were distributed and 118 valid questionnaires were recovered. Respondents are basically healthy, can take care of themselves, and can cooperate to answer questions. Demographic data: (1) age: 55–106 years old, divided into three groups: early aged group (55–5 years old), old group (60–74 years old), and old group (over 75 years old); (2) gender: 66 males and 52 females: men and women are basically equally divided; (3) education level: 5–16 years of education; (4) occupation: administrative cadres, skilled workers, workers, military personnel, and the unemployed.
2. Family pension group (home group) is the elderly living at home, including those living alone and with their children. A total of 190 questionnaires were distributed, and 176 valid questionnaires were recovered by random sampling in D city. Through validity questions, 11 invalid questionnaires and 165 valid questionnaires were deleted. Demographic data: (1) age: 55–96 years old, the same as above. The average age of this group is obviously younger than that of the social institution pension group, and the difference between them is very significant (*p* < 0.1001). (2) Gender: there are 84 males and 81 females, with almost half of them. All the respondents had no serious physical and mental diseases, and their intelligence was normal. There was no significant difference between the two groups (*p* > 0.05).

### 2.2. Research Technique

#### 2.2.1. Literature Data Method

The research consulted the national policies and regulations on the elderly and some literature on the psychology of the elderly in recent years.

#### 2.2.2. Interviewing Method

Through the collected data, interviews were conducted with the elderly and managers of 10 nursing homes and the heads of the elderly and neighborhood committees in 3 residential quarters.

#### 2.2.3. Questionnaire Survey Method

The survey was carried out by the workers of old-age care institutions and grass-roots doctors with college degree or above and special survey training. The self-made questionnaire, Geriatric Depression Scale (GDS), activities of daily living scale (ADL), and social support rating scale (SSRS) were used to investigate the two groups of elderly.

### 2.3. Statistical Method

SPSS 17.0 software was used to process the data, and the data utilization rate (%) was counted. The *X*-test was used to compare the mental health status of the elderly under different pension modes, *p* < 0.05. The difference was statistically significant.

## 3. Result

### 3.1. Comparison of Mental Health Status of the Elderly under Two Ways of Providing for the Aged

The total scores of mental health and self, emotion, and adaptation subscales in the social group were higher than those in the home group, with a significant difference (*p* < 0.05). The scores of cognitive and interpersonal subscales in the home group were higher than those in the social group, but the differences were not significant (*p* > 0.05), as given in Table 1.

### 3.2. Comparison of Health Status of the Elderly under Different Pension Models

Under the mode of family pension and social institution pension, the health status of the elderly has certain differences. Through investigation and data analysis and comparison, we find that the elderly have good memory, extensive interests, regular physical exercise, self-recognition, and good physical condition. It is obviously better than the old people in the social institution pension mode, and the data difference between them is statistically significant (*p* < 0.05). The elderly in different old-age care modes have good performance in diet and sleep, and there is no statistical difference between them (*p* < 0.05), as given in Table 2.

It can be seen from Table 1 and Table 2 that the scores of cognitive and interpersonal subscales in the family group are higher than those in the social group, but the difference is not significant (*p* < 0.05). The social institution pension mode is significantly better than the elderly, and the data difference is statistically significant (*p* < 0.05). The elderly with different pension modes perform well in diet and sleep, and the difference is not statistically significant (*p* < 0.05).

## 4. Discussion

With the transformation of the modern medical model, the definition of health not only refers to physical health but also includes mental health and good social function. Only the perfect combination of the three is the real health, especially the mental health of the elderly is more widely concerned by the society [4]. In the past, most of the research on mental health of the elderly focused on some specific elderly groups, such as retired military cadres [5], retired college elderly [6], winter swimming elderly, and so on [7]. Among the subjects, there are many younger and older people, but few older people.

With the change of family structure in China, the pace of life is accelerating, and both husband and wife lack energy and time to take care of the elderly, so some elderly people are forced or willing to enter nursing homes or nursing homes for the elderly [8]. Some of the elderly are unwilling to adapt to the new living environment, unwilling to actively communicate with others, lacking in interpersonal communication, unable to effectively solve the psychological problems encountered, and forming an unhealthy psychological state over time. The main reason is that with aging, the functions of various organs of the body decline and diseases increase, which will more or less affect behavioral ability, depression, and cognitive function, and then affect the whole mental health [9]. It can be seen from this study that the mental health status of the elderly in social institutions is basically similar to the above situation except that the gender difference is not significant. This shows that under different ways of providing for the aged, the mental health status of the elderly is similar and has its commonness. At the same time, in the process of communication, entertainment, and self-improvement, the elderly deepened their understanding of themselves and realized their personal values. Therefore, the emotional and self-scores of the elderly in the social group are significantly higher than those in the home group.

Compared with the home group, the elderly in the social group are less likely to have negative emotions such as loneliness, loneliness, and anxiety, and their mental health level is generally better than that in the home group. This is contrary to the survey results of Sommus Wei and others in Beijing urban area [10]. In this study, the material conditions and life care of the old-age care institutions are good, and the living needs of the residents are met, but the deep psychological needs and self-realization needs may not be met, thus affecting the mood of the elderly and lowering the mental health level. The elderly in the family pension mode are not stimulated by major unfortunate events or major changes, so their personality is relatively sound. In the survey, it was found that the elderly in old-age care institutions lacked hobbies and physical exercise, cognitive, intellectual and memory impairment, poor interpersonal communication, poor emotional state, and low happiness index of life, and some elderly people thought that society did not attach importance to the elderly group [11].

This study found that the mental health status of family based elderly is better than that of institutional elderly, which is inconsistent with the research results of Tian Ying [12] and consistent with the research of scholars such as Zhang Jing [13]. Generally speaking, the elderly with low economic income, strong dependence on family and society, and low social status are prone to feel inferior and suspicious. The higher the education level of the elderly, the higher the economic income, family status, and social status and the better the health status. This study shows that the elderly in the family pension mode have good interpersonal relationship, good cognition and intelligence, good adaptability, sound personality, and high happiness index, which are obviously better than those in the social institution pension mode, and the data difference between them is statistically significant. The most important thing is that there is a lack of intimate people to talk, interpersonal communication is reduced, and negative emotions are easy to occur. In addition, due to their lack of physical strength and less mental activity, their brain function declines, and they gradually come up with the idea of “old and useless” and passive old-age care, which shows the necessity and importance of paying attention to spiritual comfort in old-age care institutions.

Although most of the elderly also have home visits, this short-term relationship is far from meeting the needs of emotional communication between the elderly and their children, and it is difficult to maintain family relations. Therefore, it is suggested that the elderly themselves should expand interpersonal communication, adhere to regular physical exercise, cultivate hobbies, improve cultural quality, and maintain good mood. Retirement brings the loss of work role and the reduction of interpersonal communication to the elderly. The increase of leisure time increases the monotony and boredom of life, which is easy to induce the physiological and psychological problems of the elderly. Through the psychological needs questionnaire survey, it is found that the physical needs scores of the two groups are higher than the other three dimensions, indicating that the elderly are more inclined to meet the material needs between material needs and spiritual needs.

## 5. Conclusion

In the long run, it is a desirable way to provide for the aged in social institutions, and the transition from family pension to socialized pension will become the inevitable trend of the development of the future pension model in China. However, this kind of socialized pension needs not only the change of ideas of the elderly and their children but also the strong support of the government and the attention of the society. Only by combining material and spiritual support for the aged and improving the quality of spiritual and cultural life, can the elderly adapt to the transformation of pension mode as soon as possible and live happily in pension institutions.

## Figures and Tables

**Table 1:** Comparison of mental health scores of the elderly in two groups under the way of providing for the aged $\left(\bar{x}\pm s\right)$.

Dimension	Social group (*n* = 118)	Home group (*n* = 165)	*t* value	*P* value
Self	3.32 ± 0.29	3.27 ± 0.32	3.71	0.000
Mood	3.83 ± 0.41	3.06 ± 0.44	2.86	0.217
Adapt to	2.90 ± 0.62	2.81 ± 0.46	1.27	0.001
Cognition	3.06 ± 0.66	2.69 ± 0.28	3.38	0.061
Interpersonal	3.31 ± 1.88	3.07 ± 0.48	1.16	0.030
Aggregate score	16.42 ± 3.96	14.90 ± 1.95	2.07	0.038

**Table 2:** Comparison of health status of the elderly under different pension models $\left(\bar{x}\pm s\right)$.

Dimension	Social group (*n* = 118)	Home group (*n* = 165)	*t* value	*P* value
Good memory	1.36 ± 0.66	2.07 ± 0.71	0.84	0.322
Wide range of interests and hobbies	2.84 ± 0.52	2.62 ± 0.61	1.33	0.028
Eat and sleep well	3.37 ± 0.62	3.41 ± 0.92	2.86	0.031
Regular physical exercise	4.17 ± 0.55	3.99 ± 0.52	0.52	0.071
Self-recognition	2.88 ± 0.37	3.71 ± 0.28	1.74	0.063
In good health	3.39 ± 0.25	2.64 ± 0.43	1.62	0.082

## Data Availability

The data used to support the findings of this study are included within the article.
